The article "miR-3607-3p suppresses non-small cell lung cancer (NSCLC) by targeting TGFBR1 and CCNE2" was retracted in 2024. Reasons: duplicated images; overlap with earlier publications; unreliable results or conclusions; concerns about the images.

# miR-3607-3p suppresses non-small cell lung cancer (NSCLC) by targeting TGFBR1 and CCNE2

**DOI:** 10.1371/journal.pgen.1007790

**Published:** 2018-12-17

**Authors:** Peng Gao, Huan Wang, Jiarui Yu, Jie Zhang, Zhao Yang, Meiyue Liu, Yi Niu, Xiaomei Wei, Wei Wang, Hongmin Li, Yadi Wang, Guogui Sun

**Affiliations:** 1 Department of Radiation Oncology, North China University of Science and Technology Affiliated People’s Hospital, Tangshan, China; 2 Department of pathology, North China University of Science and Technology Affiliated People’s Hospital, Tangshan, China; 3 Department of Radiation Oncology, PLA Army General Hospital, Beijing, China; Beth Israel Deaconess Medical Center, UNITED STATES

## Abstract

Accumulating evidence indicates that miRNAs can be promising diagnostic and/or prognostic markers for various cancers. In this study, we identified a novel miRNA, miR-3607-3p, and its targets in non-small cell lung cancer (NSCLC). The expression of miR-3607-3p was measured and its correlation with patient prognosis was determined. Ectopic expression in NSCLC cells, xenografts, and metastasis models was used to evaluate the effects of miR-3607-3p on proliferation and migration of NSCLC. Luciferase assay and western blotting were performed to validate the potential targets of miR-3607-3p after preliminary screening by microarray analysis and computer-aided algorithms. We demonstrated that miR-3607-3p was downregulated in NSCLC tissues and that miR-3607-3p might act as an independent predictor for overall survival in NSCLC. Moreover, serum miR-3607-3p may be a novel and stable marker for NSCLC. We found that overexpression of miR-3607-3p inhibited cell proliferation, colony formation, migration and invasion, and hampered the cell cycle of NSCLC cell lines *in vitro*. Our results suggested that miR-3607-3p directly targets TGFBR1 and CCNE2. In accordance with *in vitro* studies, we confirmed that miR-3607-3p functions as a potent suppressor miRNA of NSCLC. We showed that miR-3607-3p agomir could reduce tumor growth and inhibit TGFBR1 and CCNE2 protein expression. Taken together, our findings indicate that miR-3607-3p can inhibit NSCLC cell growth and metastasis by targeting TGFBR1 and CCNE2 protein expression, and provide new evidence of miR-3607-3p as a potential non-invasive biomarker and therapeutic target for NSCLC.

## Author summary

We first showed downregulation of miR-3607-3p in NSCLC tissues and demonstrated that miR-3607-3p may act as an independent predictor of overall survival. Serum miR-3607-3p may be a novel marker of patients with NSCLC. We further found that miR-3607-3p possesses the potency to suppress NSCLC growth and metastasis and induce cell cycle arrest by regulating TGFBR1 and CCNE2. Importantly, agomiR-3607-3p could reduce tumor growth and lung and brain metastasis and inhibit TGFBR1 and CCNE2 protein expression. Our findings suggest that miR-3607-3p is a tumor suppressor in NSCLC and holds promise as a prognostic biomarker and potential therapeutic target for NSCLC.

The article "miR-3607-3p suppresses non-small cell lung cancer (NSCLC) by targeting TGFBR1 and CCNE2" was retracted in 2024. Reasons: duplicated images; overlap with earlier publications; unreliable results or conclusions; concerns about the images.

## Introduction

Lung cancer is one of the most frequently diagnosed cancers and the leading cause of cancer death in developed and developing countries [1]. It was estimated that there were 1,241,600 new cases of lung cancer in males and 583,100 in females in 2014 [1]. In China, it is estimated that approximately 733,300 new cases were diagnosed and 610,200 patients died of lung cancer in 2015 [2]. Approximately 85% of lung cancers are classified histopathologically as non-small cell lung carcinoma (NSCLC) [3]. In contrast to the steadily improving survival for most cancers, the 5-year survival of lung cancer is only 18% [4]. Poor outcomes and frequent relapses associated with lung cancer urgently demand the development of new screening and early biomarkers for the accurate and non-invasive detection of lung cancer metastasis and recurrence [5]. Since pathologically diagnosing all suspicious nodules is currently impossible, a noninvasive and easy sampling strategy that provides reliable information on the metastatic state of NSCLC is urgently required.

MicroRNAs (miRNAs) are small non-coding RNAs of 18–25 nt and inhibit mRNA translation and/or negatively regulate mRNA stability by binding to the 3’-untranslated region (3’-UTR) of target mRNAs [6]. The “seed” region of a miRNA is the most important known determinant of the miRNA’s ability to recognize its target mRNA [7]. Depending on the target mRNAs, miRNAs can act as either tumor oncogenes or tumor suppressors in cancers. Recent studies suggested that miRNAs are involved in a number of biological processes such as development, differentiation, proliferation, and apoptosis [8]. Dozens of miRNAs (such as miR-143/145, miR-21 and miR-34) play essential roles in lung tumorigenesis by regulating critical oncogenes or tumor suppressors [9–11]. Accumulating evidence has demonstrated that miRNAs play a critical role in either the progression or prognosis of NSCLC [12]. Several studies have shown that miRNAs could be used as diagnostic and prognostic biomarkers. For example, miR-195 expression was shown to be lower in NSCLC tissues and associated with poor survival [13]. In colorectal cancer, high expression of miR-135b and low expression of miR-590-5p are associated with clinical stage, progression and survival [14,15]. Nevertheless, most of these studies are sample and examined relatively limited numbers of miRNAs [12,16]. miR-3607-3p has been reported to be significantly attenuated and act as a crucial tumor-suppressive miRNA in prostate cancer [17]. On the other hand, Lin et al. showed that miR-3607-5p was upregulated in lung cancer tissues and cells and that miR-3607-5p overexpression promoted lung cancer A549 cells proliferation by inhibiting adenomatous polyposis coli (APC) [18], highlighting that different miRNAs from the same precursor may have different roles in different types of cancers. Since the mature miR-3607-3p and -5p species could origin from opposite sides of the miRNA hairpin and contain complex post-transcriptional miRNA regulation, it is possible that they play overlapping roles or possess different biological functions in NSCLC progression.

The article "miR-3607-3p suppresses non-small cell lung cancer (NSCLC) by targeting TGFBR1 and CCNE2" was retracted in 2024. Reasons: duplicated images; overlap with earlier publications; unreliable results or conclusions; concerns about the images.

Therefore, further study is necessary to elucidate this point. Furthermore, the precise molecular mechanism through which miR-3607-3p influences NSCLC progression remains largely unknown and further investigations are required. In addition, we were curious to determine if miR-3607-3p was associated with NSCLC in the same way as miR-3607-5p does. In this study, we identified a novel miRNA, miR-3607-3p, and its role in signaling pathways involved in the pathogenesis of NSCLC. This miRNA could be a promising biomarker and therapeutic target for NSCLC.

## Results

### miR-3607-3p expression in human NSCLC is decreased and associated with poor survival

To determine the potential functions of miR-3607-3p in NSCLC pathogenesis, we analyzed the expression of miR-3607-3p in 162 NSCLC tissue samples compared with their adjacent normal lung tissues. miR-3607-3p staining in NSCLC tissues was negative or weak relative to normal the adjacent normal lung tissues that exhibited light to dark staining (Fig 1). In contrast, miR-3607-3p signals were confined to scattered and positive images in lung tissues (Fig 1A and 1B). In situ hybridization showed that miR-3607-3p expression was significantly downregulated in tumor tissue samples compared with control samples, especially for NSCLC stages III and IV (Fig 1C and 1D, Table 1). In comparison, miR-3607-5p expression was significantly upregulated in 93 tumor tissue samples compared with control samples by in situ hybridization (S1 Fig). Downregulation of miR-3607-3p was associated with lymph node metastasis and NSCLC stage (Table 1). The Kaplan-Meier analysis indicated that patients with low miR-3607-3p expression had significantly shorter survival (commercial tissue microarray, n = 162; Fig 2A).

**Fig 1:** In situ hybridization to detect miR-3607-3p expression in 162 paired NSCLC and adjacent non-cancerous tissue samples. A negative or positive cytoplasmic signal for miR-3607-3p was observed in lung tissues. (A) Scrambled miRNA negative control (no expression). (B) U6 snRNA positive control (strong expression). (C) miR-3607-3p expression in adjacent normal lung tissues (strong expression). (D) miR-3607-3p expression in NSCLC tissues (left figure: low expression, middle figure: moderate expression, right figure: low expression).

The article "miR-3607-3p suppresses non-small cell lung cancer (NSCLC) by targeting TGFBR1 and CCNE2" was retracted in 2024. Reasons: duplicated images; overlap with earlier publications; unreliable results or conclusions; concerns about the images.

**Fig 2:** The relationship between miR-3607-3p expression levels in NSCLC tissues or serum and clinical significances. (A) Kaplan-Meier overall survival curves according to high and low miR-3607-3p expression in 162 patients with NSCLC. (B) Quantitation of miR-3607-3p was performed using qRT-PCR in 107 NSCLC (T) and adjacent normal (N) tissues. The fold changes were calculated by relative quantification (2^-ΔCt^, U6 as the internal control). (C-D) miR-3607-3p expression was detected in primary tumor tissues and the patients were grouped according to lymph node metastasis status (C) or clinical stages (D). (E) Kaplan-Meier curves depicting overall survival according to the expression of miR-3607-3p from the validation set. (F) The expression levels of serum miR-3607-3p in 80 NSCLC patients and 40 healthy controls were measured by qRT-PCR and normalized to U6. (G-H) Serum miR-3607-3p expression was low in patients with NSCLC, indicated by lymph node metastasis (G) and different clinical stages (H). (I) Receiver operating characteristic (ROC) curve analysis of the miR-3607-3p assay ratio for detecting NSCLC patients. *, *P* < 0.05.

**Table 1:** 3607-3p expression and clinicopathological parameters of NSCLC patients.

Characteristics	Training group (n = 162)			Test group (n = 107)		
	Low (n = 121)	High (n = 41)	*P*	Low (n = 80)	High (n = 27)	*P*
Gender						
Male	85 (70.8%)	32 (78.0%)	0.335	52 (65.0%)	18 (66.7%)	0.875
Female	36 (29.2%)	9 (22.0%)		28 (35.0%)	9 (33.3%)	
Age^a^						
<60	49 (40.8%)	11 (26.8%)	0.109	36 (45.0%)	10 (37.0%)	0.470
≥60	71 (59.2%)	30 (73.2%)		44 (55.0%)	17 (63.0%)	
Tumor size^a^						
< 5 cm	77 (63.6%)	26 (63.4%)	0.980	54 (69.2%)	19 (70.4%)	0.912
≥ 5 cm	44 (36.4%)	15 (36.6%)		24 (312.8%)	8 (29.6%)	
Tumor stage						
T1+ T2	89 (73.5%)	36 (87.8%)	0.060	61 (76.3%)	24 (88.9%)	0.160
T3+ T4	32 (26.5%)	5 (12.2%)		19 (23.7%)	3 (11.1%)	
Histological type						
Adenocarcinoma	69 (57.0%)	18 (43.9%)	0.145	42 (52.5%)	14 (51.9%)	0.954
Squamous cell carcinoma	52 (43.0%)	23 (56.1%)		38 (47.5%)	13 (48.1%)	
Histological grade^a^						
Well/moderate	88 (72.7%)	27 (65.9%)	0.402	44 (62.0%)	20 (74.1%)	0.261
Poor/NS	33 (27.3%)	14 (34.1%)		27 (38.0%)	7 (25.9%)	
Lymph node metastasis^a^						
Negative	53 (54.6%)	30 (75.0%)	0.027	44 (54.3%)	23 (85.2%)	0.005
Positive	44 (45.4%)	10 (25.0%)		36 (45.7%)	4 (14.8%)	
Clinical stages^a^						
I + II	61 (52.1%)	33 (80.5%)	0.001	44 (54.3%)	24 (88.9%)	0.002
III + IV	56 (47.9%)	8 (19.5%)		36 (45.7%)	3 (11.1%)	

^a^Numbers do not equal to the total number due to missing data.

qRT-PCR showed that miR-3607-3p levels in NSCLC tissue samples were markedly lower than in normal lung tissue samples (n = 107; Fig 2B), particularly in samples from patients with lymph node metastasis and advanced clinical stages of NSCLC (Fig 2C and 2D, Table 1). Kaplan-Meier survival analysis also revealed that miR-3607-3p downregulation was associated with poor prognosis in patients with NSCLC (specimens from patients, n = 107; Fig 2E). Multivariate Cox regression analysis showed that the miRNA signatures were an independent prognostic factor for OS of NSCLC (Table 2).

The article "miR-3607-3p suppresses non-small cell lung cancer (NSCLC) by targeting TGFBR1 and CCNE2" was retracted in 2024. Reasons: duplicated images; overlap with earlier publications; unreliable results or conclusions; concerns about the images.

**Table 2:** Multivariate cox regression analysis of factors associated with overall survival in NSCLC.

Variable	Training group (n = 162)			Test group (n = 107)		
	95%CI	*RR*	*P*	95%CI	*RR*	*P*
Sex (male vs. female)	0.516–1.672	0.929	0.805	0.516–5.712	1.717	0.378
Age (≤60 vs.>60 years)	0.781–2.204	1.312	0.305	0.653–2.479	1.272	0.480
Tumor size (≤5cm vs.>5 cm)	0.765–2.346	1.340	0.306	0.599–2.468	1.216	0.588
Tumor stages (T1+T2 vs. T3+ T4)	0.361–1.290	0.682	0.240	0.615–3.057	1.371	0.440
Histological type (Adenocarcinoma vs. Squamous cell carcinoma)	0.353–1.147	0.636	0.133	0.713–8.233	2.423	0156
Histologic grade (Well/ moderate vs. Poor/NS)	0.576–1.682	0.984	0.954	0.397–1.828	0.852	0.681
Lymph node metastasis (negative vs. positive)	1.060–4.234	2.119	0.034	1.027–6.312	2.546	0.044
Clinical stages (I + II vs. III + IV)	1.031–4.497	2.153	0.041	1.038–7.698	2.827	0.042
miR-3607-3p expression levels (Low vs. High)	0.207–0.713	0.278	0.002	0.041–0.921	0.194	0.039

qRT-PCR showed that serum expression levels of miR-3607-3p were significantly lower in NSCLC patients than in normal controls (Fig 2F, Table 3). Serum miR-3607-3p expression levels were negatively associated with lymph node metastasis and advanced clinical stages of NSCLC (Fig 2G and 2H, Table 3). The area under the curve (AUC) for plasma miR-3607-3p was 0.810, indicating that there was an obvious significance in NSCLC diagnosis by serum miR-3607-3p (Fig 2I).

**Table 3:** Serum expression levels of miR-3607-3p and clinicopathological characteristics in patients with NSCLC.

Characteristics	miR-3607-3p expression status		
	Low (n = 40)	High (n = 40)	*P*
Gender			
Male	26 (65.0%)	27 (67.5%)	0.813
Female	14 (35.0%)	13 (22.5%)	
Age^a^			
<60	19 (47.5%)	16 (40.0%)	0.499
≥60	21 (52.5%)	24 (60.0%)	
Tumor size			
< 5 cm	27 (67.5%)	31 (77.5%)	0.317
≥ 5 cm	13 (22.5%)	9 (22.5%)	
Tumor stage			
T1+ T2	28 (70.0%)	35 (87.5%)	0.056
T3+ T4	12 (30.0%)	5 (12.5%)	
Histological type			
Adenocarcinoma	27 (67.5%)	21 (52.5%)	0.171
Squamous cell carcinoma	13 (22.5%)	19 (47.5%)	
Histological grade^a^			
Well/moderate	28 (70.0%)	25 (64.1%)	0.577
Poor/NS	12 (30.0%)	14 (35.9%)	
Lymph node metastasis			
Negative	17 (42.5%)	31 (77.5%)	0.001
Positive	23 (57.5%)	9 (22.5%)	
Clinical stages			
I + II	18 (45.0%)	30 (75.0%)	0.006
III + IV	22 (55.0%)	10 (25.0%)	

^a^Numbers do not equal to the total number due to missing data.

The article "miR-3607-3p suppresses non-small cell lung cancer (NSCLC) by targeting TGFBR1 and CCNE2" was retracted in 2024. Reasons: duplicated images; overlap with earlier publications; unreliable results or conclusions; concerns about the images.

### miR-3607-3p shows suppressive effects on NSCLC cell growth and metastasis

Among the six NSCLC cell lines and normal human embryo lung fibroblast cell line (MRC-5), the H157 and H292 cell lines had the lowest expression of miR-3607-3p (Fig 3A) and the highest metastatic potential (S2 Fig); therefore, they were selected for the overexpression experiment. To further investigate the role of miR-3607-3p in the regulation of NSCLC cell proliferation, colony formation, invasion, and migration, H157 and H292 cells were transfected with an miR-3607-3p mimic and miR-3607-3p levels were examined using qRT-PCR. The efficiency of transfection was verified as a significant increase in miR-3607-3p expression in H157 and H292 cells by qRT-PCR (Fig 2B and S3A Fig). High exogenous expression of miR-3607-3p remarkably inhibited proliferation, colony formation, migration, and invasion of H157 and H292 cells (Fig 2C–2E and S3B–S3D Fig). Similarly, we observed that the exogenous high expression level of miR-3607-3p remarkably inhibited proliferation and invasion of normal human embryo lung fibroblast MRC-5 cell line (S4A–S4C Fig). To explore the possible mechanisms underlying the inhibitory effect on cell growth by overexpression of miR-3607-3p, a cell cycle analysis was performed. Upon upregulation of miR-3607-3p, the percentages of H157 and H292 cells in G0/G1 phase increased compared with the percentages measured in controls (Fig 3F and S3E Fig), indicating that overexpression of miR-3607-3p resulted in G1 phase arrest in NSCLC cells.

**Fig 3:** miR-3607-3p overexpression inhibited cell proliferation, colony formation, and migration in NSCLC cell lines. (A) RNA level of miR-3607-3p in six NSCLC cell lines. (B) Quantitation of miR-3607-3p level after the transfection of miR-3607-3p mimic (50 ng/L) in H157 cell lines. (C) Cell growth curve measured by MTS after the transfection of miR-3607-3p mimic (50 ng/L) in H157 cell lines; all OD 570 values were normalized to the starting point (0 hour). (D) Representative images and quantitative results of colony formation were obtained after transfection with miR-3607-3p mimic (50 ng/L) in H157 cell lines. (E) Representative images and quantitative results of the Transwell assay were obtained after transfection with miR-3607-3p mimic (50 ng/L) in H157 cell lines. (F) miR-3607-3p induced cell cycle arrest at G1/S phase. Data are presented as means ± standard deviation from triplicate experiments. *, *P* < 0.05.

The article "miR-3607-3p suppresses non-small cell lung cancer (NSCLC) by targeting TGFBR1 and CCNE2" was retracted in 2024. Reasons: duplicated images; overlap with earlier publications; unreliable results or conclusions; concerns about the images.

Next, we transfected NSCLC cells with inhibitors of miR-3607-3p to confirm the opposite results of mimic transfection (Fig 4A and S5A Fig). As expected, downregulation of miR-3607-3p using the inhibitors could enhance the malignant phenotype of A549 and H1299 cells *in vitro*, including cell growth (Fig 4B and S5B Fig) and colony formation (Fig 3C and S5C Fig), as well as cell migration and invasion (Fig 3D and S5D Fig). We further observed that forced expression of miR-3607-3p could decrease the number of cells in G1 phase and increase the numbers of cells in S phase (Fig 3E and S5E Fig). Hence, miR-3607-3p downregulation could be promoting cell proliferation.

**Fig 4:** Repression of miR-3607-3p expression significantly promoted cell growth, colony formation, and migration in A549 cells. (A) Quantitative measurement of miR-3607-3p level after the transfection of miR-3607-3p inhibitor (100 ng/L) in A549 cell lines. (B) Cell growth curve measured by MTS after transfection with miR-3607-3p inhibitor (100 ng/L) in A549 cell lines; all OD 570 values were normalized to the starting point (0 hour). (C) Representative images and quantitative results of colony formation were obtained after transfection with miR-3607-3p inhibitor (100 ng/L) in A549 cell lines. (D) Representative images and quantitative results of the Transwell assay were obtained after the transfection of miR-3607-3p inhibitor (100 ng/L) in A549 cell lines. (E) miR-4317 induced cell cycle arrest at G1/S phase. Data are presented as means ± standard deviation from triplicate experiments. *, *P* < 0.05.

### miR-3607-3p targets TGFBR1 and CCNE2 to suppress proliferation and metastasis

To explore the mechanism through which miR-3607-3p regulates NSCLC cell progression, we searched for potential downstream targets of miR-3607-3p using several bioinformatics methods, including miRWalk, TargetScan, and miRDB (Fig 5A). Several candidate genes involved in proliferation, cycling and invasion-metastasis were identified by gene ontology (GO) terms and qRT-PCR. We found that TGF-β receptor 1 (TGFBR1) and cyclin E2 (CCNE2), two key proteins involved in TGF-β signaling and the cell cycle pathway, appeared to be potential targets of miR-3607-3p (Fig 5B). To verify whether TGFBR1 and CCNE2 are direct targets of miR-3607-3p, we transfected an miR-3607-3p mimic into cells and observed that this could markedly down-regulate the mRNA and protein levels of *TGFBR1* and *CCNE2* in H157 and H292 cells, respectively (Fig 5C and 5D). We also transfected NSCLC cells with inhibitors of miR-3607-3p to confirm the results of mimic transfection. As expected, downregulation of miR-3607-3p using inhibitors could enhance the *TGFBR1* and *CCNE2* mRNA and protein levels in A549 and H1299 cells (Fig 5E and 5F). We next applied the dual-luciferase reporter method to reveal the regulation of miR-3607-3p by TGFBR1 and CCNE2. The fragments containing the miR-3607-3p binding sequence or mutated sequence in the 3’UTR regions of *TGFBR1* and *CCNE2* were cloned into the pmiR-RB-REPORT vector luciferase reporter. These reporter constructs were co-transfected with miR-3607-3p mimic or miR-NC into H157 and H292 cells, and the luciferase activities were subsequently measured. The miR-3607-3p mimic significantly suppressed the luciferase activity of pmiR-RB-REPORT-TGFBR1 or CCNE2-3’UTR (Fig 5G and 5H), while miR-NC had no inhibitory effect on pmiR-RB-REPORT TGFBR1 or CCNE2-3’UTR. The miR-3607-3p inhibition of pmiR-RB-REPORT-TGFBR1 and CCNE2-3’UTR was sequence-specific because the luciferase activities of pmiR-RB-REPORT-TGFBR1 or CCNE2-mut did not decrease in the presence of miR-3607-3p. Taken together, these results suggest that miR-3607-3p can directly target the 3’-UTR of *TGFBR1* and *CCNE2*.

The article "miR-3607-3p suppresses non-small cell lung cancer (NSCLC) by targeting TGFBR1 and CCNE2" was retracted in 2024. Reasons: duplicated images; overlap with earlier publications; unreliable results or conclusions; concerns about the images.

**Fig 5:** *TGFBR1* and *CCNE2* are two direct target genes of miR-3607-3p. (A-B) *TGFBR1* and *CCNE2* were identified as potential regulatory targets of miR-3607-3p by considering the downregulation genes using prediction tools and the qRT-PCR method. (C-D) The expression levels of *TGFBR1* and *CCNE2* mRNA and protein were measured by qRT-PCR and western blot analysis using GAPDH as the loading control after transfection of miR-3607-3p mimic in H157 and H292 cell lines, respectively. (E-F) The expression levels of *TGFBR1* and *CCNE2* mRNA and protein were measured by qRT-PCR and western blot analysis using GAPDH as the loading control after transfection of miR-3607-3p inhibitors in A549 and H1299 cell lines, respectively. (G-H) Dual-luciferase reporter assay. The relative luciferase activity was normalized to the Renilla luciferase activity after co-transfection of cells with miR-3607-3p mimic and pmiR-RB-REPORT construct containing WT or MUT TGFBR1 and CCNE2 3’-UTR region in H157 and H292 cell lines. Data are presented as means ± standard deviation from triplicate experiments. *, *P* < 0.05.

A rescue experiment was performed to confirm that TGFBR1 or CCNE2 was the functional target of miR-3607-3p in H157 and H292 cells. The evidence was obtained from the observation that the *TGFBR1* or *CCNE2* mRNA and protein (endogenous) in the two cell lines were diminished by mimic transfection and recovered by transfection of both pEGFP-N1-TGFBR1 or CCNE2 expression constructs, respectively (Fig 6A–6C). The results showed that migration and invasion created by mimic transfection were reversed by transfection of both expression constructs (Fig 6D and 6E).

The article "miR-3607-3p suppresses non-small cell lung cancer (NSCLC) by targeting TGFBR1 and CCNE2" was retracted in 2024. Reasons: duplicated images; overlap with earlier publications; unreliable results or conclusions; concerns about the images.

**Fig 6:** Rescue assays were performed to confirm that TGFBR1 and CCNE2 are the functional targets of miR-3607-3p. (A-C) The mRNA and protein levels of *TGFBR1* and *CCNE2* in H157 and H292 cell lines with co-transfection of miR-3607-3p mimic and pEGFP-C1 plasmid containing *TGFBR1* and *CCNE2* CDS sequence. (D-E) Transwell assay of co-transfection cell with miR-3607-3p mimic and TGFBR1 and CCNE2 plasmid. Data are presented as means ± standard deviation from triplicate experiments. *, *P* < 0.05.

### miR-3607-3p suppresses tumor growth and metastasis *in vivo*

Finally, we evaluated the effects of miR-3607-3p on the growth and metastasis of NSCLC in nude mice. A549 cells were transfected with either a lentiviral expression vector to knock down miR-3607-3p or a negative control lentiviral vector. The downregulation of miR-3607-3p in the A549 cells following lentiviral infection was verified by qRT-PCR (Fig 7A). Then, we injected these A549 cells subcutaneously in BALB/c nude mouse to induce tumors. Beginning on day 7 after injection, the tumor lengths and widths were measured every 5 days for 40 days. The tumor growth curve revealed a significantly higher growth rate in the miR-3607-3p-downregulated group compared with the control group (Fig 7B). Subsequently, the tumors were dissected and the exact dimensions and weights were evaluated. Compared with the control group, the tumors in the miR-3607-3p-downregulated group were larger (Fig 7C and 7D).

**Fig 7:** miR-3607-3p suppressed tumor growth and metastasis *in vivo*. (A) Levels of miR-3607-3p in stable miR-3607-3p knockdown A549 cells (Lenti-inhibitor) and control A549 cells (Lenti-vector). (B-D) Stable miR-3607-3p knockdown A549 cells were subcutaneously injected into nude mice to form solid tumors and representative images of tumor volumes and weights were analyzed by *in vivo* luciferase imaging on the endpoint day (n = 5 for each group). (E-G) The numbers of metastatic nodules were observed and quantified in the lungs and brain of mice treated with stable miR-3607-3p knockdown A549 cells or control vector cells by tail vein injection. (H-J) The A549 cells were subcutaneously injected into nude mice to form solid tumors and were treated with miR-3607-3p agomir or miR agomir NC (n = 5 for each group). A 10-nmol miR-3607-3p agomir and the miRNA negative control in 0.1 ml saline buffer were locally injected into the tumor masses once every 5 days for 6 weeks. (K) Immunohistochemistry of Ki67, TGFBR1, and CCNE2 in tumor tissues dissected from nude mice treated with miR-3607-3p agomir or miR angomir NC. (L) TGFBR1 and CCNE2 protein expression measured by immunohistochemistry in 162 NSCLC samples and association with lung cancer survival. (M-N) Spearman correlation analysis of the negative correlation between the expression of miR-3607-3p and TGFBR1/ CCNE2. *, *P* < 0.05.

The article "miR-3607-3p suppresses non-small cell lung cancer (NSCLC) by targeting TGFBR1 and CCNE2" was retracted in 2024. Reasons: duplicated images; overlap with earlier publications; unreliable results or conclusions; concerns about the images.

Luciferase-labeled cells (10^6^) were injected intravenously in the tail vein of mice and the animals were sacrificed 6 weeks later. Luciferase activity was used to evaluate the tumor burden in the lung and brain. The lung metastasis burden was significantly higher in the mice injected with miR-3607-3p-knockdown cells compared with the control group (Fig 7E and 7F). As expected, knockdown of miR-3607-3p significantly increased the brain metastasis through tail vein injection (Fig 7E and 7G). All these results obtained for the mouse models suggest that miR-3607-3p plays important roles in NSCLC growth and metastasis *in vivo*, particularly in lung and brain metastasis. To determine whether miR-3607-3p could inhibit the growth of NSCLC in nude mice, we established nude mouse tumorigenic and metastatic model using A549 cells, as above. After 7 days, miR-3607-3p agomir or miR agomir NC were directly injected into the subcutaneous tumor every 5 days for 35 days. The tumor volume was measured every 5 days until day 42. The tumor volume and weight of mice treated with miR-3607-3p agomir were significantly greater than those of mice treated with miR agomir NC (Fig 7H–7J). This result indicated that miR-3607-3p significantly inhibits the tumorigenicity of A549 cells in the nude mouse model.

In addition, the proliferative activities of the tumor cells were assessed by immunohistochemistry for Ki-67 in FFPE tissues of xenograft tumors. The Ki-67 staining was decreased in tumors from the miR-3607-3p agomir group (Fig 7K). Moreover, a distinct decrease in TGFBR1 or CCNE2 expression was observed in IHC slices of the miR-3607-3p agomir group compared with the expression observed for the miR agomir NC group (Fig 7K). TGFBR1 or CCNE2 expression was significantly higher in tumor tissues than in adjacent non-tumor tissues (n = 70; Fig 7L). miR-3607-3p expression was inversely correlated to the expression of TGFBR1 and CCNE2 in NSCLC specimens (n = 70; Fig 7M and 7N).

## Discussion

MicroRNAs have recently been demonstrated to contribute to carcinogenesis and the progression of various cancers and may provide new therapeutic strategies such as the use of biomarkers and therapeutic targets [19,20]. In this study, we found that miR-3607-3p, an intronic miRNA located at chromosomal position 5q14.3, is frequently downregulated in human NSCLC specimens. Our analyses suggest that low miR-3607-3p expression can be an important biomarker for discriminating between normal lung and tumor tissues. Correlations with clinicopathological parameters suggest that downregulation of miR-3607-3p is associated with tumor progression in NSCLC. Low miR-3607-3p expression was significantly associated with NSCLC of higher stages and with lymph node metastasis. These results are consistent with recent findings indicating that expression levels of tumor-suppressing miRNAs are often downregulated in NSCLC.

The article "miR-3607-3p suppresses non-small cell lung cancer (NSCLC) by targeting TGFBR1 and CCNE2" was retracted in 2024. Reasons: duplicated images; overlap with earlier publications; unreliable results or conclusions; concerns about the images.

Many miRNAs have been associated with tumor-suppressive effects in NSCLDC and other types of cancer. For example, miR-195 expression has been shown to be lower in tumor tissues and was associated with clinical stages of NSCLC [13]. miR-720 acts as a tumor suppressor by inhibiting cell migration and invasion, and was found to be downregulated in primary breast carcinoma [20]. miRNAs have also been extensively investigated as prognostic factors [21]. Zhou et al. also demonstrated that high expression of miR-574-5p in serum was an independent factor of poor prognostic in patients with SCLC [22]. The present study suggests that miR-3607-3p is an independent prognostic factor for OS in NSCLC. In addition, our results showed that lower expression of miR-3607-3p might be associated with poor overall survival in NSCLC. Poor prognosis of patients with early-stage lung cancer is associated with lymph node metastasis and distant metastasis at the time of presentation [23]. Regarding the role of miR-3607 in other cancer types, Saini et al. [17] showed that the miR-3607-3p region is frequently deleted in prostate cancer, highlighting potential tumor-suppressive roles of this family. A recent study showed that CirclRAK3 sponges miR-3607-3p and facilitates breast cancer metastatic spread [24]. In hepatocellular carcinoma, low expression of miR-3607-3p predicts poor prognosis [25]. Collectively, these findings suggest that miR-3607-3p may be a novel biomarker for NSCLC prognosis and diagnosis. However, Lin et al. [18] reported that miR-3607-5p had opposite roles compared with miR-3607-3p. Since the sequences of the two miRNAs are different, it is possible that they possess different roles. Indeed, it is accepted that the mature miRNA -3p and -5p species originate from the opposite sides of the same miRNA hairpin and have complex post-transcriptional miR-3607 regulation. Therefore, both species would regulate a unique set of targets and possess very different biological functions. Hence, further study is necessary to elucidate this point. Indeed, miR-3607-3p has been reported to be significantly attenuated in prostate cancer [17]. On the other hand, miR-3607-5p was upregulated in lung cancer and miR-3607-5p overexpression promoted lung cancer A549 cells proliferation [18]. Those two studies support the results of the present study, but additional research is still necessary to examine this dual effects of the same miRNA.

The article "miR-3607-3p suppresses non-small cell lung cancer (NSCLC) by targeting TGFBR1 and CCNE2" was retracted in 2024. Reasons: duplicated images; overlap with earlier publications; unreliable results or conclusions; concerns about the images.

Endogenous circulating miRNAs could be significant for the diagnosis, prognosis, and metastasis of cancer. Our results suggest that serum miR-3607-3p levels might be useful in delineating lung cancer stages because of decreasing expression of miR-3607-3p in higher-stage cancers. Indeed, the AUC value was 0.81 in NSCLC patients compared with normal controls. These findings indicate that miR-3607-3p levels could hold great diagnostic potential, with high sensitivity and specificity. In other words, serum miR-3607-3p level could be a good noninvasive biomarker for NSCLC diagnosis. Tumor-derived miRNAs were first described in plasma by Mitchell et al. [26]. Accumulating evidence suggests the potential of miRNAs in the early detection of several malignancies such as lung cancer [27], breast cancer [28], and gastric cancer [29]. In addition, serum miR-146a has been reported in papillary thyroid carcinoma [30], lung cancer [31], and gastric cancer [32], which is associated with diagnosis and can be used for early detection of tumors.

Differences in miRNA expression in tumor samples do not necessarily alter the function of tumor cells. Our *in vitro* results suggested that miR-3607-3p mimic suppressed the proliferation, colony formation, and migration abilities of NSCLC cells, while transfection of miR-3607-3p inhibitor had the opposite effects. Lower levels of miR-3607-3p not only enhanced cell viability but also promoted colony formation and cell migration. Importantly, data from the present study revealed that upregulation of miR-3607-3p reduced tumor growth and metastasis *in vivo* by delivery of the agomir into cancer cells and the tail vein in nude mice. Recent studies have indicated that miRNAs play a potential role as tumor suppressors in NSCLC and other types of cancers [33,34]. Joshi et al. demonstrated that miR-148a might act as a tumor suppressor and that the miRNA inhibited the migration and invasion of the A549 NSCLC cell line [5]. Yu et al. conducted an *in vitro* study of NSCLC cell lines and provided evidence that cell proliferation, migration and invasion could be evaluated by the transfection of miR-520a-3p [35]. Similarly, the roles of miR-675-5p in regulating tumor growth and metastasis *in vivo* have been demonstrated in previous studies [27]. In gastric cancer, forced expression of miR-26b led to inhibition of GC cell migration and invasion *in vitro* and lung metastasis formation *in vivo* [36]. Conversely, miR-151-5p could promote tumor growth and lung metastasis of SC-M1 cells *in vivo* through downregulation of p53 protein expression in NSCLC [37]. All these results support our findings that miR-3607-3p functions as a tumor suppressor gene. miR-3607-3p may be the basis of new approaches to cancer therapy via the mechanisms of its regulation of tumors.

The article "miR-3607-3p suppresses non-small cell lung cancer (NSCLC) by targeting TGFBR1 and CCNE2" was retracted in 2024. Reasons: duplicated images; overlap with earlier publications; unreliable results or conclusions; concerns about the images.

Although the mechanism by which miRNAs alter gene expression remains controversial, most studies have suggested that miRNAs are primarily processed by the RNA-mediated interference machinery to trigger partial or complete target gene mRNA degradation [38]. Our bioinformatics analysis revealed that miR-3607-3p could bind to the 3′UTR of TGFBR1 and CCNE2, repressing their expression. TGFBR1 is an important element of the TGF-β/SMAD signaling pathway, which has emerged as a central mediator of cancer progression because of its ability to regulate cell growth, differentiation, and migration [39]. The TGF-β pathway controls a plethora of cellular responses and plays a crucial role in tumorigenesis as either tumor promoter or suppressor [40]. Regarding tumor promotion, the TGF-β pathway could stimulate cell invasion by inducing epithelial-mesenchymal transition (EMT) and ultimately promote metastasis in multiple tumors [41–43]. TGF-β binding to TGFBR2 leads to phosphorylation and activation of TGFBR1 by TGFBR2. With the help of SARA, Smad2/3 is phosphorylated by TGFBR1. Then, they form a heterotrimeric complex with Smad4 and translocate into the nucleus to regulate gene transcription [44]. Yang et al. demonstrated that miR-140-5p possesses the potency to suppress hepatocellular carcinoma growth and metastasis by regulating TGFBR1 and FGF9 [45]. Studies have also shown that repression of TGFBR1 inhibits the cell proliferation of lung cancer and cell migration and invasion of breast cancer [46,47]. Previous studies highlighted the role of TGFBR1 in NSCLC [48,49].

CCNE2 is a well-known cyclin involved in the progression of the cell cycle, specifically the G1/S transition. CCNE2 is also involved in the development of NSCLC [2,50,51]. In this study, we conducted FACS analysis to further confirm how miR-3607-3p acts as a negative regulator of the cell cycle and found that increasing the expression of this miRNA resulted in significant G0/G1 arrest and S phage reduction. Cyclin E proteins play critical roles in G1 phase and in the G1-S phase transition with cyclin-dependent kinase 2 (CDK2) [2]. Overexpression of CCNE1 and CCNE2 has been reported in many types of human cancers. Recent data clearly showed that restoration of miR-144-5p function in bladder cancer cells inhibited the expression of both CCNE1 and CCNE2 and significantly induced G1 arrest in bladder cancer cells [52]. These results suggest that miR-3607-3p might inhibit NSCLC growth and metastasis partly by targeting TGFBR1 and CCNE2. The Ki-67 staining intensities were decreased in the tumors from the miR-3607-3p-overexpressing group. Our results further showed stronger TGFBR1 and CCNE2 staining in xenograft tumors of the miR-3607-3p agomir group than in tumors of the NC group, indicating that the proliferation of tumor cells was increased by the down-expression of miR-3607-3p. The present study is not without limitations. TGFBR1 and CCNE2 were evaluated in the tumor tissue and normal adjacent tissue samples in the mouse model. Since the tumors cells are of human origin and the ‘normal adjacent tissue’ is of mouse origin, differing reactivity of the antibodies with human and mouse proteins could be concerning. Finally, miR-3607-5p should be tested along miR-3607-3p within the same sets of experiments.

The article "miR-3607-3p suppresses non-small cell lung cancer (NSCLC) by targeting TGFBR1 and CCNE2" was retracted in 2024. Reasons: duplicated images; overlap with earlier publications; unreliable results or conclusions; concerns about the images.

In conclusion, our results strongly suggest that miR-3607-3p is downregulated in NSCLC tissues and miR-3607-3p might act as an independent predictor for overall survival in NSCLC. Our results also suggest that serum miR-3607-3p could be a novel and stable biomarker for NSCLC. Furthermore, we found that miR-3607-3p possesses the potency to suppress NSCLC growth and metastasis, and to induce cell cycle arrest by regulating TGFBR1 and CCNE2. Our findings suggest that miR-3607-3p functions as a tumor suppressor in NSCLC and holds promise as a prognostic biomarker and potential therapeutic target for NSCLC.

## Methods

### Tissue samples

An organized chip array including 162 non-metastatic NSCLC tissue samples and non-neoplastic lung tissue samples was purchased from Outdo Biotech (HlugA180Su02 and HLug-Squ150Sur-02, Shanghai, China; http://www.superchip.com.cn/). A total of 107 paired frozen paraffin NSCLC tissue samples and matched adjacent non-cancerous tissue samples were obtained from the North China University of Science and Technology Affiliated People’s Hospital; the tissues were collected between 2009 and 2013. In addition, the serum samples from 80 patients with NSCLC and 40 healthy controls were obtained from the North China University of Science and Technology Affiliated People’s Hospital; serum samples were stored at -80°C. For studies using human data, the study was approved by ethics committee of the North China University of Science and Technology Affiliated People’s Hospital. (approval number: RH-2017-006) and written informed consent was obtained from all participants.

The article "miR-3607-3p suppresses non-small cell lung cancer (NSCLC) by targeting TGFBR1 and CCNE2" was retracted in 2024. Reasons: duplicated images; overlap with earlier publications; unreliable results or conclusions; concerns about the images.

### Cell culture

The human lung adenocarcinoma cell lines A549, NCI-H1299, NCI-H157, ANIP-973, NCI-H292, and PC-9 were obtained from the Cell Culture Center of Peking Union Medical College (Beijing, China). The human embryonic kidney (HEK) 293T cell line was obtained from the American Tissue Culture Collection (Manassas, VA). The NSCLC cell lines were cultured in RPMI-1640 medium. HEK 293 T cells were maintained in DMEM supplemented with 10% fetal bovine serum (Gibco BRL, Grand Island, NY) in a humidified atmosphere of 5% CO_2_ at 37°C. The human fetal lung fibroblast cell line (MRC-5) was cultured in Minimum Essential Medium (MEM) containing non-essential amino acids, Earle’s salts, and L-glutamine supplemented with 10% fetal bovine serum and 1% antibiotic-antimycotic solution (containing 100 U/mL penicillin, 100 μg/mL streptomycin, and 0.25 μg amphotericin), and was maintained in a humidified air atmosphere with 5% CO_2_ at 37°C.

### In situ hybridization of miR-3607-3p

In situ hybridization (ISH) was performed according to the manufacturer’s instructions (Roche Molecular Systems, Pleasanton, CA, USA). The miR-3607-3p and miR-3607-5p probes (5’*-*CATCAGAAAGCGTTTACAGT*-*3’ and 5’*-*GCAUGUGAUGAAGCAAAUCAGU*-*3’) were tagged with 3’ and 5’ digoxigenin (Redlandbio.biomart.cn, Guangzhou, China). U6 snRNA (5’*-*CACGAATTTGCGTGTCATCCTT*-*3’) and scrambled probes (5*′*-GTGTAACACGTCTATACGCCCA*-*3′) were used as positive and negative controls, respectively. The probe-target complex was detected using an antidigoxigenin-alkaline phosphates conjugate and nitro-blue tetrazolium and 5-bromo-4-chloro-3’-indolyphosphate as the chromogen. The signals were classified according to cytoplasmic miR-3607-3p intensity as: negative: negative or faint expression in most cells; low expression: low expression in most cells or moderate expression in <50% of the cells; and high expression: moderate to strong expression in most cells. At least five random fields were evaluated by assessors blinded to grouping and clinical features.

### miRNA transfection

All endogenous mature miRNA mimics, inhibitors and agomirs were purchased from RiboBio (Guangzhou, China). Transfection was performed according to the manufacturer’s protocols. miRNA mimics (50 nmol/L), miRNA inhibitors (100 nmol/L), and miRNA negative controls (NC) (100 nmol/L) were transfected into the cells using Lipofectamine 2000 (Invitrogen, Carlsbad, USA) according to the manufacturer’s instructions. After 48 h of transfection, cells were used for further experiments.

The article "miR-3607-3p suppresses non-small cell lung cancer (NSCLC) by targeting TGFBR1 and CCNE2" was retracted in 2024. Reasons: duplicated images; overlap with earlier publications; unreliable results or conclusions; concerns about the images.

### Plasmid construction

pDonR223-TGFBR1 and pDonR223-CCNE2 plasmids carrying the human TGFBR1 and CCNE2 genes were purchased from Changsha Axybio Bio-Tech Co., Ltd (Changsha, China, S1–S5 Files). The complete coding sequences of human TGFBR1 and CCNE2 were amplified from the pDonR223-TGFBR1 and pDonR223-CCNE2 plasmids. TGFBR1 and CCNE2 products and pEGFP-N1 plasmid were digested with *Xho I* and *Hind III*, and the fragments were purified and ligated with T4 DNA ligase. The ligated products were transformed into TOP10 competent cells. The positive clones were named pEGFP-N1-TGFBR1 and pEGFP-N1-CCNE2.

### Quantitative real-time polymerase chain reaction

To evaluate the expression of miR-3607-3p, TGFBR1, CCNE2, and other genes, total RNA was used for reverse transcription (RT) and quantitative polymerase chain reaction (qRT-PCR) was performed on a Step One Plus real-time system (AB Applied Biosystems, Carlsbad, CA). U6 and GAPDH were used as internal controls. All the primers used in this study are listed in S6 File.

### Target prediction and luciferase reporter assay

Bioinformatics analysis was performed using the following software: miRWalk, miRanda, and TargetScan. The 3’-UTR of human *TGFBR1* and *CCNE2* was amplified from human genomic DNA and individually inserted into the pmiR-RB-REPORT (Ribobio, Guangzhou, China, S7-8 file) using the *XhoI* and *NotI* sites. Similarly, the fragment of *TGFBR1* and *CCNE2* 3’-UTR mutant was inserted into the pmiR-RB-REPORT control vector at the same sites. For reporter assays, NSCLC cells were co-transfected with wild type reporter plasmid and miR-3607-3p mimics. Firefly and Renilla luciferase activities were measured in cell lysates using the Dual-Luciferase Reporter Assay system. Luciferase activity was measured 48 h post-transfection using the dual-glo luciferase reporter system according to the manufacturer’s instructions. Firefly luciferase units were normalized against Renilla luciferase units to control for transfection efficiency.

### *In vitro* cell proliferation assay

For cell proliferation assays, cells were seeded on a 96-well plate (5×10^3^ per well) and cell proliferation was determined by MTS (3-(4,5-dimethylthiazol-2-yl)-5-(3–carboxymethoxyphenyl)-2-(4-sulfophenyl)-2H-tetrazolium) according to the manufacturer’s instructions. MTS solution was added (20 μl/well) to each well and incubated at 37°C for 2 h. The optical density of each sample was immediately measured using a microplate reader (BioRad, Hercules, CA, USA) at 570 nm.

### Colony formation assay

Cells were transfected with miR-3607-3p mimic or miR mimic NC, miR-3607-3p inhibitor or miR inhibitor NC, as described above. After 24 h, the transfected cells were trypsinized, counted and re-plated at 1×10^3^ cells/10-cm dish. After 10 days, colonies resulting from the surviving cells were fixed with 3.7% methanol, stained with 0.1% crystal violet and counted. Colonies containing at least 50 cells were scored. Each assay was performed in triplicate.

The article "miR-3607-3p suppresses non-small cell lung cancer (NSCLC) by targeting TGFBR1 and CCNE2" was retracted in 2024. Reasons: duplicated images; overlap with earlier publications; unreliable results or conclusions; concerns about the images.

### Transwell migration/invasion assay

*In vitro* cell migration assays were performed as described previously using Trans-well chambers (8 μM pore size; Costar). Cells were allowed to grow to ~75–80% confluency and serum-starved for 24 h. After detachment with trypsin, cells were washed with PBS and resuspended in serum-free medium. Next, 100 μl of cell suspension (5×10^4^ cells/mL) were added to the upper chamber. Complete medium was added to the bottom wells of the chambers. The cells that had not migrated after 24 h were removed from the upper face of the filters using cotton swabs, but the cells that had migrated were fixed with 5% glutaraldehyde solution to determine the number of migratory cells. The lower surfaces of the filters were stained with 0.25% Trypan Blue. Images of six random ×10 fields were captured from each membrane and the number of migratory cells was counted. The assay was performed in triplicate for each experimental condition and the mean values were used for analysis. Similar inserts coated with Matrigel were used to evaluate the cell invasive potential in the invasion assay.

### Flow cytometry analysis

Fluorescence-activated cell sorting (FACS) analysis was performed 48 h after transfection. The cells were harvested, washed with cold PBS, and fixed into 70% ethanol at -20°C for 24 h, stained with 50 μg/mL propidium iodide (PI) (4ABio, China), and analyzed using a FACS Calibur flow cytometer (BD Bioscience, MA). The results were analyzed using the ModFit software (BD Bioscience, USA). Assays were conducted three independent times.

### Western blot analysis

For western blot analysis, RIPA buffer containing protease inhibitors and phosphatase inhibitors (Roche) was used to prepare whole-cell lysates. Equal amounts of proteins were separated by SDS-polyacrylamide gel electrophoresis (SDS-PAGE) and transferred to PVDF membranes (Millipore). After blocking with 5% bovine serum albumin (BSA), the membranes were probed with anti-TGFBR1, CCNE2, and anti-GAPDH (ab31013, ab32103, and ab8425; Abcam, Cambridge, UK), followed by incubation with a horseradish peroxidase-conjugated secondary antibody goat-anti-mouse IgG (1:2000) and goat-anti-rabbit IgG (1:3000). Proteins were visualized using Image Reader LAS-4000 (Fujifilm) and analyzed using the Multi Gauge V3.2 software.

### Generation of stable cell lines

Recombinant lentiviral vectors containing miR-3607-3p knockdown and irrelevant sequences were purchased from XIEBHC Biotechnology (Beijing, China, S9 File). In addition to the lentivirus expression vectors, there was a luciferase and puromycin reporter gene driven by the EF1α promoter to indicate the infection efficiency in a timely manner. To construct the lentiviral vectors, the precursor sequence for miR-3607-3p and the irrelevant sequence (negative control) were inserted into pHBLV-U6-MCS-EF1α-Luc-T2A-puromycin lentiviral vectors. The recombinant lentiviruses were packaged by co-transfection of HEK-293T cells with pSPAX2 and pMD2.G with the LipoFiter reagent. The supernatants with lentivirus particles were harvested at 48 and 72 h after transfection and filtered through 0.45-μm cellulose acetate filters (Millipore, USA). Recombinant lentiviruses were concentrated by ultracentrifugation. To establish stable cell lines, NSCLC cells were transduced with lentivirus with a MOI of approximately 5 in the presence of 5 μg/ml polybrene. The supernatant was removed after 24 h and replaced with fresh complete culture medium. Infection efficiency was confirmed by RT-PCR 96 h after infection. The cells were selected with 2 μg/ml puromycin for 2 weeks.

The article "miR-3607-3p suppresses non-small cell lung cancer (NSCLC) by targeting TGFBR1 and CCNE2" was retracted in 2024. Reasons: duplicated images; overlap with earlier publications; unreliable results or conclusions; concerns about the images.

### Tumorigenicity and metastasis assay *in vivo*

For studies using animal data, all experiments were performed according to the Regulations for the Administration of Affairs Concerning Experimental Animals of 1988, issued by the State Scientific and Technological Commission for China. And these experiments were approved by the Institutional Animal Care and Use Committee of the North China University of Science and Technology Affiliated People’s Hospital (approval number: RM-2017-035). The effects of miR-3607-3p on the tumorigenic and metastatic potential of NSCLC cells were analyzed in subcutaneous and systemic metastasis in vivo models via right hip subcutaneous tissue injection and tail vein injection, respectively. For the subcutaneous model, 4-6-week-old BALB/c nude mice were injected subcutaneously in the right hip with 1×10^6^ transfected cells. For the experimental metastasis in vivo model, transfected cancer cells (1×10^6^ in 100 μl of HBSS) were directly injected into the tail vein. Six weeks later, tumor colonies in subcutaneous tissue were observed by HE staining and histology examination. Bioluminescence images were collected to assess the growth and metastasis of implanted tumor cells. To quantify the in vivo bioluminescence signals, mice were anesthetized with isoflurane before in vivo imaging. A D-luciferin solution (in vivo imaging solutions, PerkinElmer, 150 mg/kg in PBS) was injected intravenously for both orthotopic and systemic xenografts. Bioluminescence images were acquired with the IVIS Spectrum imaging system (Perkin-Elmer Life Sciences, Waltham, MA, USA) 2–5 min after injection. The captured images were quantified using the Living Image Software package (Perkin Elmer/ Caliper Life Sciences) by measuring the photon flux (photons/s/cm2/steradian) within a region of interest (ROI) drawn around the bioluminescence signal.

The article "miR-3607-3p suppresses non-small cell lung cancer (NSCLC) by targeting TGFBR1 and CCNE2" was retracted in 2024. Reasons: duplicated images; overlap with earlier publications; unreliable results or conclusions; concerns about the images.

### Agomir treatment

The agomir and miRNA negative control were synthesized by Ribobio (Guangzhou, China) and used according to the manufacturer’s instructions. A 10-nmol miR-3607-3p agomir as well as the miRNA negative control in 0.1 ml of saline buffer were locally injected into NSCLC cell-forming tumor mass once every 5 days for 6 weeks. After treatment, the NSCLC cell-forming tumors were tested by immunohistochemistry. The tumor size was monitored by measuring the length (L) and width (W) with calipers every 5 days. The volumes were calculated using the formula (L × W^2^)/2. Mice were sacrificed by cervical dislocation on day 42. The tumors were excised and snap-frozen for protein and RNA extraction.

### Immunohistochemistry

The sections were de-paraffinized and boiled in 10 mM citrate buffer (pH 6.0) for antigen retrieval. Endogenous peroxidase was blocked by 3% H_2_O_2_. Slides were blocked in serum, incubated with the indicated antibodies at 4°C overnight, incubated with anti-rabbit secondary antibody, and visualized with diaminobenzadine (Sigma). A negative control experiment was also performed. IHC staining images were captured at 200× under a microscope (Olympus).

### Statistical analysis

All continuous data were expressed as means ± standard deviation. Error bars represented the standard errors of the means. Student’s t-test, χ^2^ test and repeated measures ANOVA were used to determine statistical significance, as appropriate. The log-rank test was used to analyze the effect of clinical variables and miRNAs on the overall survival (OS) of patients. Multivariate Cox regression models were used to assess factors associated with overall survival in NSCLC. Cox regression analysis was used to evaluate the independent prognostic value of the miR-3607-3p signature, with age, gender, T stage, histological type, N stage, clinical stage, and the miRNA signature used as covariates. Receiver operating characteristic (ROC) curves and the area under the ROC curve (AUC) were used to assess the feasibility of using serum miRNA as a diagnostic tool for detecting NSCLC. *P* < 0.05 was considered statistically significant. Statistical analyses were performed using SPSS 16.0 (IBM, Armonk, NY, USA).

### Ethics approval and consent to participate

This study was reviewed and approved by the Ethics Committee of North China University of Science and Technology Affiliated People’s Hospital.

The article "miR-3607-3p suppresses non-small cell lung cancer (NSCLC) by targeting TGFBR1 and CCNE2" was retracted in 2024. Reasons: duplicated images; overlap with earlier publications; unreliable results or conclusions; concerns about the images.

## Supporting information

S1 Fig In situ hybridization to detect miR-3607-5p expression in 93 paired NSCLC and adjacent non-cancerous tissues. (A) miR-3607-5p expression in adjacent normal lung tissues (none or low expression). (B) miR-3607-5p expression in NSCLC tissues (strong expression).
(JPG)

S2 Fig The metastatic ability of 6 NSCLC cell lines has been measured by Transwell assay. (A-B) Representative images and quantitative results of Transwell assay were obtained after the transfection of miR-3607-3p mimic in NSCLC cell line. *, *P* < 0.05.
(JPG)

S3 Fig miR-3607-3p overexpression inhibited cell proliferation, colony formation, and migration. (A) Quantitation of miR-3607-3p levels after the transfection of miR-3607-3p mimic in H292 cell lines. (B) Cell growth curve measured by MTS after the transfection of miR-3607-3p mimic in H292 cell lines; all OD 570 values were normalized to the starting point (0 hour). (C) Representative images and quantitative results of colony formation were obtained after the transfection of miR-3607-3p mimic in H292 cell lines. (D) Representative images and quantitative results of the Transwell assay were obtained after transfection of miR-3607-3p mimic in A549 cell lines. (E) miR-3607-3p induced cell cycle arrest at G1/S phase. Data are presented as the means ± standard deviation from triplicate experiments. *, *P* < 0.05.
(JPG)

S4 Fig miR-3607-3p overexpression inhibited cell proliferation, migration and invasion in MRC-5 cell line. (A) Quantitation of miR-3607-3p level after the transfection of miR-3607-3p mimic in MRC-5 cell lines. (B) Cell growth curve measured by MTS after the transfection of miR-3607-3p mimic in MRC-5 cell line; all OD 570 values were normalized to the starting point (0 hour). (C) Representative images and quantitative results of the Transwell assay were obtained after transfection of miR-3607-3p mimic in MRC-5 cell line. *, *P* < 0.05.
(JPG)

S5 Fig Repression of miR-3607-3p expression significantly promoted cell growth, colony formation, and migration in H1299 cells. (A) Quantitative results of miR-3607-3p level obtained after the transfection of miR-3607-3p inhibitor in H1299 cell lines. (B) Cell growth curve measured by MTS after the transfection of miR-3607-3p inhibitor in H157 cell lines; all OD 570 values were normalized to the starting point (0 hour). (C) Representative images and quantitative results of colony formation were obtained after the transfection of miR-3607-3p inhibitor in H1299 cell lines. (D) Representative images and quantitative results of the Transwell assay were obtained after transfection of miR-3607-3p inhibitor in H1299 cell lines. E. miR-3607-3p induced cell cycle arrest at G1/S phase. Data are presented as the mean values ± SD from triplicate experiments. *, *P* < 0.05.
(JPG)

S1 File The TGFBR1 carrier map. (ZIP)

S2 File The plasmid construction of TGFBR1. (ZIP)

S3 File The plasmid construction of TGFBR1. (ZIP)

S4 File The CCNE2 carrier map. (ZIP)

S5 File The plasmid construction of CCNE2. (ZIP)

S6 File Specific primers used in this study (5’-3'). (ZIP)

S7 File The vector construction 3'UTR region of TGFBR1. (ZIP)

S8 File The vector construction 3'UTR region of CCNE2. (ZIP)

S9 File Sequencing result of miR-3607-3p knockdown. (ZIP)

S1 Data Numerical data underlying of the Fig 2. (XLSX)

S2 Data Numerical data underlying of the Fig 3. (XLSX)

S3 Data Numerical data underlying of the Fig 4. (XLSX)

S4 Data Numerical data underlying of the Fig 5. (XLSX)

S5 Data Numerical data underlying of the Fig 6. (XLSX)

S6 Data Numerical data underlying of the Fig 7. (XLSX)
